# HIF-1*α* Ameliorates Diabetic Neuropathic Pain via Parkin-Mediated Mitophagy in a Mouse Model

**DOI:** 10.1155/2022/5274375

**Published:** 2022-08-16

**Authors:** Jian He, Zaisheng Qin, Xin Chen, Wanyou He, Donglin Li, Lei Zhang, Yue Le, Qingming Xiong, Bin Zhang, Hanbing Wang

**Affiliations:** ^1^Department of Anesthesiology, The First People's Hospital of Foshan, Foshan City, China; ^2^Department of Anesthesiology, Nanfang Hospital, Southern Medical University, Guangzhou City, China; ^3^Department of Critical Medicine, Foshan Hospital of Traditional Chinese Medicine, Foshan City, China

## Abstract

Mitochondrial dysfunction, which can be regulated by mitophagy, plays a central role in diabetic neuropathic pain (DNP). Mitophagy that was involved in nerve damage-induced neuropathic pain has been reported. Hyperglycemia and cellular hypoxic were the two main characters of diabetes. Hypoxia-inducible factor 1*α* subunit (HIF-1*α*) plays a vital role in mitochondrial homeostasis under hypoxia. However, it remains unclear whether mitophagy was changed and could be regulated by HIF-1*α* in DNP. In this study, the results showed that mitophagy was activated and HIF-1*α* was upregulated in the spinal cord of diabetic mice. HIF-1*α* agonist dimethyloxalylglycine (DMOG) could further elevate HIF-1*α* and Parkin protein, enhance mitophagy, decrease mitochondrial dysfunction, and hyperalgesia. Furthermore, Park2 (encoding Parkin) knockout aggravated hyperalgesia and mitochondrial dysfunction in diabetic mice. Furthermore, mitophagy could not be activated and induced by HIF-1*α* agonist DMOG in Park2^−/−^ diabetic mice. In this study, we first demonstrated that HIF-1*α* could upregulate mitophagy in the spinal cord of mice with DNP through modulating the Parkin signaling pathway, promoting new insights into the mechanisms and research of treatment strategies for patients with DNP.

## 1. Introduction

Diabetes mellitus is the leading cause of secondary complications such as diabetic nephropathy, retinopathy, and diabetic neuropathy [1–3]. The major cause of diabetes mellitus is hyperglycemia and nonenzymatic glycation reaction that, when not treated, leads to the complications, including neuropathic pain [4–6]. Neuropathic pain is one of the most common complications in diabetic patients, yet the implementation of effective therapeutic strategies is challenging [7, 8]. Diabetic neuropathic pain (DNP) is characterized by spontaneous and stimulus-evoked pain, such as hyperalgesia and allodynia [7, 9]. The mechanism underlying the pathogenesis of DNP remains unknown [8, 9]. Hyperglycemia is considered the leading pathogenic factor in the development of neuropathic pain [10]. However, even under careful control of glycemia, chronic complications like neuropathy, retinopathy, or nephropathy may not be prevented, delayed, or attenuated [11]. These evidences suggest that organ injury caused by hyperglycemia cannot be reversed by strictly controlling blood glucose. The pathogenesis of hyperglycemia-related diabetic neuropathy is primarily attributed to oxidative stress and mitochondrial dysfunction [12, 13]. However, antioxidant treatment can only provide a limited therapeutic effect on DNP. This implies that antioxidants can only scavenge or antagonize existing reactive oxygen species (ROS) induced by oxidative stress but cannot prevent the generation of ROS from damaged mitochondria, which are the main source of intracellular ROS in diabetes [14]. Increasing evidence shows that hyperglycemia-induced mitochondrial dysfunction plays a central role in the development of DNP [7, 15]. In particular, neurons are a kind of high energy-consuming cells and rely on the intact and function mitochondrial to provide energy. Therefore, it is remarkably important to search for new therapeutic and preventive strategies to improve neuron mitochondrial dysfunction and maintain intracellular homeostasis.

Autophagy is a degrading mechanism for the recycling and turnover of damaged organelles and macromolecules in cells [16]. Mitophagy is a kind of selective autophagy in which injured mitochondria are degraded to maintain proper mitochondrial function [16]. Recently, emerging evidence suggests that mitophagy plays a pivotal role in human diseases, including neuropathic pain [17, 18]. Furthermore, mitophagy is also involved in the development of hyperglycemia-induced heart and kidney damage in the animal model [19, 20]. In addition, abnormal mitophagy was one of the main factors of neurodegenerative diseases [21, 22], including Parkinson's disease, Alzheimer's disease, and Huntington's disease. However, it remains unknown whether mitophagy involves DNP and the underlying mechanism.

Hypoxia-inducible factor 1 (HIF-1) induced mitophagy was the main mechanism to eliminate dysfunction mitochondrial and maintain cellular homeostasis under hypoxia [23, 24]. Hyperglycemia can promote oxidative phosphorylation and increase oxygen consumption in mitochondria, resulting in cellular hypoxia and a subsequent active downstream signal pathway [12, 25]. High glucose was reported to directly induce hypoxia in glomerular endothelial, vascular endothelial cells, and neurons in vitro [26, 27]. Moreover, HIF-1*α* (a functional subunit of HIF-1) was altered in the heart, kidney [27], and retinal tissues [28] of diabetes and can regulate these organ complications induced by hyperglycemia through mitophagy. In addition, a recent report suggests that HIF-1*α* expression was increased in peripheral nerve fibers in a patient with diabetes [29]. These data imply the relationship between HIF-1*α* and diabetic complications, but the exact molecular mechanism is unclear.

Park2 is a frequently mutated gene that was first found in Parkinson's disease [30]. Parkin, which is encoded by Park2, is an E3 ubiquitin ligase and can mark specific proteins with ubiquitin for degradation through the ubiquitin-proteasome system [31]. Growing evidence has shown that Parkin plays a key role in neuroprotection through mitophagy [32, 33]. Furthermore, Parkin was involved in hyperglycemia-induced heart [34] and kidney dysfunction [35]. In addition, recent studies have suggested that Parkin-mediated mitophagy was regulated by HIF-1*α* under hypoxia [36, 37]. However, the relationship between Parkin and HIF-1*α* under the hyperglycemia condition is still unclear.

In the present study, we investigated the roles of HIF-1*α* in the regulation of mitochondrial function and pain hypersensitivity and the potential mechanisms in a mouse model of type I diabetes induced by streptozotocin (STZ). Our study demonstrated that HIF-1*α* could alleviate DNP through Parkin-mediated mitophagy in the spinal cord of a mouse model.

## 2. Materials and Methods

### 2.1. Animals

All animal experimental procedures were approved by the Animal Use and Care Committee for Research and Education of the First People's Hospital of Foshan (Foshan, PR China). Adult male C57BL/6 mice (8 weeks old, 20–24 g, center of laboratory animal science of Guangdong, China) were used in animal experiments. The mice were housed at a constant room temperature of 21 ± 2°C and a relative humidity of 55 ± 5% under a 12 h light/dark cycle with ad libitum access to food and water. Park2 knockout (KO) mice were obtained from Professor Tao Li. All efforts were made to minimize the pain and fear of the animal.

### 2.2. Streptozotocin- (STZ-) Induced Diabetes Mellitus

Diabetes mellitus was established by a single intraperitoneal (i.p.) injection of streptozotocin (150 mg/kg body weight, Sigma-Aldrich) freshly dissolved in citrate buffer (pH = 4.5, 0.1 M). The control mice were injected with equivalent vehicle (i.p.). The mice with plasma glucose concentration higher than >16.7 mmol/L 3 days after STZ injection were defined as hyperglycemia [35, 38]. The mice were removed from the study without hyperglycemia 3 days after STZ injection. All animals were retested for blood glucose and body weight once per week throughout the experiments.

### 2.3. Experimental Protocol

The present study was divided into two parts. In experiment 1, we observed changes in the behavior and mitophagy in diabetic mice and the influence of HIF-1*α* on DNP. In experiment 2, we explored the effects of Parkin-mediated mitophagy on HIF-1*α* regulated DNP.

In experiment 1, thirty-two C57BL/6 mice were randomly divided into four groups (*n* = 8 per group): group NC (the sham group), group DP (the diabetes group), group DM (the DP+HIF-1 agonist treatment group), and group ME (the DP+HIF-1 antagonists treatment group). The HIF-1 agonist dimethyloxalylglycine (DMOG, 250 mg/kg, i.p.) or the antagonist methoxyestradiol (2ME, 15 mg/kg, i.p.) was injected for 7 consecutive days from the fifth week after STZ injection. The mechanical withdrawal threshold (PWT) and thermal withdrawal latency (TWL) were measured at 1 d before and 7, 14, 21, and 28 d after STZ injection and 1, 3, 5, and 7 d after injection of HIF-1 agonist or antagonist. The L4–L6 spinal cord segments were collected at 7 days after injection of HIF-1 agonist or antagonist for further examination.

In experiment 2, twenty-four Park2 KO mice were randomly divided into three groups (*n* = 8 per group) by random number table: the NC group (sham group), DP group (diabetic group), and DM group (treatment group DP+HIF-1 agonist). Twenty-four wild-type (WT) mice were also randomly divided into three groups as the same method. The HIF-1 agonist was injected as in experiment 1. The behavior test was consistent with experiment 1.

### 2.4. Behavior Tests

Before behavioral tests, mice were individually taken to the test compartments and allowed to adjust to the environment for 30 min. The PWT was assessed using an electronic Von Frey algesimeter (Bioseb, Chaville, France) according to the previous study [39]. The nociceptive stimulation to which the paw withdrawal responded was automatically turned off and the mechanical force that evoked the response was recorded. Every mouse was subjected to three tests, with 15 min intervals, and the average force was taken as the PWT. The TWL was used to evaluate thermal sensitivity. Mice were placed on a hot (53°C) transparent resin plate and the time that the mice spent licking their hind paws or jumping was recorded. Every mouse was tested three tests, with an interval of 10 min, and the average time spent was taken as the TWL. A cut-off point of 30 s was set to avoid burn injuries.

### 2.5. Western Blot and Antibodies

After the last behavioral tests, mice were deeply anesthetized with pentobarbital (100 mg/kg, i.p.) and transcardially perfused with phosphate-buffered saline (PBS, pH 7.4) for 10 min. The L4-L6 spinal cord segments were quickly dissected and homogenized in iced lysis buffer (pH 8.0, 150 mM NaCl, 50 mM Tris-HCl, 1% IGEPAL, 1 mM EDTA, 0.5% Na-deoxycholate, and 0.1% SDS) contained protease inhibitors (Sigma-Aldrich, Milan, Italy) and incubated on ice for 30 min. The mixture tissue samples were then centrifuged at 14,000 × g for 15 min at 4°C, and the supernatants were collected. Protein concentrations were determined using a BCA protein assay kit (Beyotime, Jiangsu, China). Subsequently, the sample was mixed with loading buffer and heated at 95°C for 8 min. For western blot analysis, an equal amount of total protein was separated by 8%-12% SDS-PAGE gels and transferred to PVDF membranes (Immobilon-P, Sigma-Aldrich, Milan, Italy). The PVDF membranes were blocked using 5% nonfat milk for 1 hour at room temperature and then incubated with the primary antibody overnight at 4°C. After rinsing thrice, the membranes were incubated with HRP-conjugated goat anti-rabbit IgG secondary antibodies (1 : 5000, Abcam, UK) for 2 h at room temperature. Peroxidase activity was visualized using the ECL Western Blotting Detection Kit (Bio-Rad, Shanghai, China). Protein intensity was measured and analyzed using Bio-Rad Quantity One software (Bio-Rad Company, CA, USA). The following primary antibodies and dilutions were employed: anti-LC3 (1 : 1000, Cell Signaling Technology, USA), anti-Beclin1 (1 : 1000, Cell Signaling Technology, USA), anti-p62/SQSTM1(1 : 1000, Cell Signaling Technology, USA), anti-TOM20 (1 : 1,000, BD, USA), anti-parkin (1 : 1,000; Thermo Invitrogen, USA), anti-HIF-1*α* (1 : 1000, Abcam, USA), and anti-GAPDH (1 : 1000, Affinity, China).

### 2.6. Immunohistochemistry and Immunofluorescence Analysis

The lumbar enlargement (L4-L6) was harvested as above, transferred to 4% paraformaldehyde, and stored at 4°C. Transverse spinal cord paraffin sections (at the thickness of 6 *μ*m) were dewaxed with xylene and then rehydrated in a sequence of 100%, 95%, 75%, and 50% ethanol. Immunohistochemistry was performed according to the previous study [40]. Antigens were recovered by heating them in a microwave oven (microwave method) at 90°C for 15 min. The sections were then blocked with 0.3% hydrogen peroxide (*v*/*v*) hydrogen peroxide and incubated in a wet box for 10 minutes. Sections were incubated with a monoclonal antibody against HIF-1*α* (1 : 200, Ab1, Abcam, USA) overnight in a humid dark chamber at 4°C. After washing with PBS, the slices were incubated with biotinylated anti-rabbit IgG and a streptavidin–peroxidase complex (Vector Laboratories, Inc., Burlingame, CA, USA) for 10 min at room temperature. The immunostaining of sections was visualized using diaminobenzidine (DAB), and the nucleus was counterstained with hematoxylin.

According to our previous study on immunofluorescence staining [41], after antigen retrieval, sections were blocked with 10% normal goat serum for 60 min and then incubated with the following primary antibodies: anti-LC3 (1 : 200, Cell Signaling Technology, USA) and anti-TOM20 (1 : 200, Millipore, USA), at 4°C overnight. After a series of PBS rinses, the slices were incubated for 2 h with Dylight 594 (1 : 100, Abcam, USA) or Dylight488-conjugated goat anti-rabbit IgG (1 : 100, Abcam, USA) in the PBS buffer. The slices were counterstained with 4′,6-diamidino-2′-phenylindole (DAPI) and were visualized with a fluorescence microscope (Olympus, Tokyo, Japan).

### 2.7. Measurement of Mitochondrial Membrane Potential

According to the manufacturer's instructions, mitochondrial membrane potential (MMP) was detected using a JC-1 kit (MAK 147, Beyotime, China). The lumbar enlargement tissue was washed twice with 1640 complete medium and was repeatedly cut into small pieces. The small pieces of tissue were digested with 0.25% trypsin at 37°C for 20 min. The digested spinal cord tissue was transformed into a cell suspension through a 70 *μ*m cell sieve. The cell suspension was obtained at 1000 rpm and centrifuged for 5 min to collect cell precipitation. Cells were incubated with the JC-1 agent in the dark for 20 minutes at 37°C. The precipitated cells were washed twice with PBS, and then the cells were resuspended with an appropriate amount of PBS for flow cytometry. The relative MMP was calculated based on red/green fluorescence ratio, as described previously (16).

### 2.8. Measurement of Intracellular Reactive Oxygen Species

Intracellular ROS levels were measured using the fluorescent probe 2′,7′-dichlorofluorescin diacetate (DCFH-DA, Beyotime, China). Cell suspension was produced according to the MMP examination method and then incubated with DCFH-DA at 37°C for 20 minutes. Fluorescence intensity was analyzed by flow cytometry using excitation/emission wavelengths of 488/525 nm.

### 2.9. Electron Microscopy

Mice were deeply anesthetized with pentobarbital sodium (100 mg/kg) and perfused with ice PBS into the left ventricle to flush the blood. The L4-6 spinal cord segment was taken out, and was quickly cut into 1 mm^3^ small pieces on the ice, put into 2.5% glutaraldehyde buffer EP tube, and fixed in 4°C refrigerator for 24 h. The sample was fixed with 1% Russian acid for 2 hours and then dehydrated with 30%, 50%, 70%, 80%, 90%, and 100% acetone step by step.

The dehydrated samples were embedded in epon and cut into 60 nm thick sections. The slices were stained with0.4% uranyl acetate and 2% lead citrate. Ultrastructural organelle images were obtained by an electron microscope (Hitachi, Tokyo, Japan) in a blinded manner.

### 2.10. Statistical Analysis

SPSS 16.0 software (SPSS Inc., Chicago, IL, USA) was used to analyze the data. The measurement data are presented as the means ± S.E. (standard error of the mean). The statistical differences between groups were analyzed using a one-way analysis of variance (ANOVA), followed by Bonferroni Student's *t*-test. Repeated measurement data from behavioral tests were analyzed using a two-way analysis of variance followed by Bonferroni Student's *t*-test. Differences of *P* < 0.05 were considered to be significant.

## 3. Results

### 3.1. The Level of HIF-1*α* Was Increased in Diabetic Mice

To explore whether HIF-1*α* was involved in the development of diabetic neuropathic pain, HIF-1*α* expression was measured by western blotting and immunostaining. As shown in Figure 1(a), the level of HIF-1*α* was increased in the spinal cord of STZ-induced diabetic mice compared to normal mice, which indicated HIF-1*α* was induced by hyperglycemia. HIF-1*α* agonist DMOG and antagonist 2-ME were injected into the diabetic mice for further exploring the role of HIF-1*α* in the development of DNP. The western blot results showed that DMOG treatment could further increase the expression of HIF-1*α* in diabetic mice, but 2-ME inhibited the increase of HIF-1*α* induced by hyperglycemia (Figures 1(a) and 1(b)). These data were also verified by immunohistochemistry. As shown in Figures 1(c) and 1(d), the number of HIF-1*α*-positive cells in the spinal dorsal horn of diabetic mice was more than that in the control mice. DMOG treatment could further increase the number of HIF-1*α*-positive cells, but 2-ME treatment decreased the number of HIF-1*α*-positive cells in the spinal dorsal horn of diabetic mice. These results demonstrated that DMOG and 2-ME treatment could alter HIF-1*α* expression in the spinal cord of diabetic mice.

### 3.2. Overexpression of HIF-1*α* Alleviated Hyperalgesia in Diabetic Mice

To investigate the role of HIF-1*α* on the DNP, we first established the DNP model in mice using STZ injection. Blood glucose levels of mice were measured weekly throughout the study. Three days after STZ injection, the mice presented hyperglycemia and maintained high blood glucose throughout the experiment (Figure 2(a)). Both HIF-1*α* agonist DMOG and inhibitor 2-ME did not affect the blood glucose of diabetic mice (Figure 2(a)).

Mice gradually decreased the mechanical pain threshold and thermal withdrawal latency from the second week to the fourth week after STZ injection (Figures 2(b) and 2(c)). These results indicated that the mice develop DNP following STZ injection. To verify the hypothesis that HIF-1*α* could regulate DNP, we investigated the effect of DMOG and 2-ME on DNP in mice. DMOG treatment significantly mitigated mechanical hyperalgesia in diabetic mice, while 2-ME exacerbates mechanical hyperalgesia in diabetic mice compared to nonsupplemented diabetic mice. Consistent with this, DMOG treatment alleviated thermal hyperalgesia and 2-ME increased thermal hyperalgesia in diabetic mice (Figures 2(b) and 2(c)). Taken together, these results indicated that HIF-1*α* overexpression could mitigate STZ-induced hyperalgesia in the mouse model.

### 3.3. Overexpression of HIF-1*α* Improved Mitochondrial Dysfunction in the Spinal Cord of Diabetic Mice

Mitochondrial dysfunction plays a central role in the development of DNP. To assess the mitochondrial function in the spinal cord in mice with DNP, ROS generation and mitochondrial membrane potential were measured in this study. The mitochondrial membrane potential was lower in diabetic mice than that in nondiabetic mice (Figure 3(a)). Consistent with this, the amount of ROS was higher in the diabetic mice than that in the nondiabetic mice measured by JC-1 fluorescence (Figure 3(b)). These results showed that the mice with DNP occurred mitochondrial dysfunction in the spinal cord. To determine whether HIF-1*α* alters the mitochondrial function of the spinal cord in mice with DNP, we used DMOG and 2-ME treatment diabetic mice for 7 consecutive days. DMOG inhibited ROS accumulation and loss of mitochondrial membrane potential induced by hyperglycemia (Figures 3(a) and 3(b)). Conversely, 2-ME aggravated the ROS accumulation and further decreased mitochondrial membrane potential (Figures 3(a) and 3(b)). These results indicated that overexpression of HIF-1*α* could improve mitochondrial dysfunction of the spinal cord in diabetic mice.

### 3.4. Overexpression of HIF-1*α* Increased Mitophagy in the Spinal Cord of Diabetic Mice

Mitophagy was the most important mechanism to maintain mitochondrial homeostasis and was evaluated in this study. Microtubule-associated protein light chain 3 (LC3) is a crucial protein to form the autophagosome and exists in two forms. A cytosolic LC3 (LC3-I) is an unconjugated form and can convert to LC3-II by conjugation to phosphatidylethanolamine. Because LC3-II is combined with autophagosomes and is related to autophagy, one method of evaluating autophagy is to examine the conversion of LC3 (LC3-I to LC3-II). However, due to several problems, the LC3-I and LC3-II ration may not be appropriate and, instead, the amount of LC3-II can be compared between samples [42]. Beclin 1 protein is another essential factor in the initiation step of autophagosome formation [43]. The increased expression of Beclin 1 indicated active autophagy. The p62/SQSTM1 protein, which binds to the LC3 associated with autophagy, is a vital autophagy substrate and can be efficiently degraded by autophagy [44]. Thus, the p62 protein can accumulate when autophagy is blocked [44].

In the present study, the levels of LC3 II and Beclin1 of the spinal cord in diabetic mice were higher than those in the control mice (Figure 4(a)). However, the level of P62 was lower of the spinal cord in diabetic mice compared to the controlled mice (Figure 4(a)). DMOG can further increase the expression of LC3 II and Beclin1 and promote the degradation of the P62 protein in the spinal cord of DNP mice (Figure 4(a)). In contrast, 2-ME can inhibit the expression of LC3 II and Beclin1 and decrease the degradation of P62 in DNP mice (Figure 4(a)). These results indicated that autophagy was induced in the spinal cord in diabetic mice, and overexpression of HIF-1*α* could further enhance autophagy. Otherwise, there are several types of autophagy according to the contents of autophagosomes, including endoplasmic reticulum autophagy, Golgi autophagy, and mitochondrial autophagy. Therefore, we used double immunofluorescence staining to further demonstrate the change in autophagy in diabetic mice. The TOM20 protein was located in the outer membrane of mitochondrial and was used as a mitochondrial marker. In this study, the numbers of immunoreactive cells against TOM20 and LC3-II were higher in the spinal cord of diabetic mice than those of controlled mice by double immunofluorescence staining (Figure 4(b)). Treatment with DMOG treatment could further increase the number of cells against TOM20 and LC3-II in diabetic mice (Figure 4(b)). However, treatment with the HIF-1*α* antagonist 2-ME decreased the number of immunoreactive cells against TOM20 and LC3-II compared to non-treatment diabetic mice (Figure 4(b)). These results further demonstrated that mitophagy was induced in the spinal cord of diabetic mice. Electron microscopy was also used to observe the mitochondrial structure and further verify mitophagy. Electron microscopic images showed an increase in mitochondrial autophagosomes in the spinal cord in diabetic mice compared to control mice. DMOG could further increase the number of mitochondrial autophagosomes in diabetic mice, but 2-ME decreased the number of mitochondrial autophagosomes (Figure 4(c)). Together, these data demonstrated that mitophagy was induced and HIF-1*α* overexpression can further increase spinal mitophagy in diabetic mice.

### 3.5. Park2 Deficiency Accelerated the Development of Neuropathic Pain in Diabetic Mice

HIF-1*α* can alleviate hyperalgesia through mitophagy in diabetic mice; the exact underlying molecular mechanism remains unclear. To explore the effect of Park2 on the DNP, Park2 KO mice were used to establish the diabetic model. There was no significant difference in blood glucose between WT and Park2 KO mice on the basal line and after STZ injection (Figure 5(a)). These results suggested that the Park2 knockout did not alter the blood glucose of mice. Furthermore, Park2 KO mice did not present any change in PWT and TWL at baseline compared to Park2 WT mice. This data suggested Park2 deletion did not alter the baseline pain threshold. The PWT and TWL were decreased in the second week in WT diabetic mice, but it was reduced in the first week in the Park2 KO diabetic mice (Figures 5(b)–5(e)). Moreover, the PWT and TWL were lower in Park2 KO diabetic mice than that in WT diabetic mice on 7, 14, 21, and 28 days after STZ injection (Figures 5(b) and 5(e)). These results indicated that Park2 knockout accelerated the development of neuropathic pain in diabetic mice. To investigate the role of HIF-1*α* on the Park2 KO and WT DNP mice, DMOG treatment was administered from 29 days to 35 days after STZ injection. PWT and TWL increased at 3, 5, and 7 after injection of DMOG in WT diabetic mice, but not in Park2 KO diabetic mice (Figures 5(b)–5(g)). These results indicated that overexpression of HIF-1*α* alleviates DNP through the Parkin protein.

### 3.6. Park2 Knockout Aggravated Hyperglycemia-Associated Mitochondrial Dysfunction in Diabetic Mice

To evaluate the effect of Park2 knockout on mitochondrial function, we tested the MMP and ROS content in the spinal cord of Park2 KO diabetic mice. The ROS level was higher in the spinal cord of Park2 KO diabetic mice than in WT diabetic mice (Figures 6(a) and 6(b)). DMOG could inhibit the increased generation of ROS in WT diabetic mice but not in KO diabetic mice (Figures 6(a) and 6(b)). Similar to these, the MMP was lower in the spinal cord of Park2 KO diabetic mice than that in WT diabetic mice (Figures 6(c) and 6(d)). DMOG could partly reverse the decrease in hyperglycemia-induced MMP in WT mice, but not in Park2 KO diabetic mice (Figures 6(c) and 6(d)). These results suggested that Park2 KO aggravated hyperglycemia-induced mitochondrial dysfunction, and HIF-1*α* improved mitochondrial dysfunction depending on the Parkin protein.

### 3.7. Mitophagy Could Not Be Induced by Hyperglycemia in the Spinal Cord in Park2-Deficient Mice

We examine the effect of Park2 deletion on mitophagy in the spinal cord in DNP mice. There was no significant difference in LC-II, Beclin1, and P62 expressions in the spinal cord of Park2 KO and WT nondiabetic mice (Figures 7(a)–7(d)). These results suggest that Park2 depletion did not alter the basal autophagy of mice. Furthermore, the LC3-II, Beclin1, and P62 protein also did not change in Park2 KO diabetic mice compared to Park2 KO nondiabetic mice (Figures 7(a)–7(d)). This result indicated that hyperglycemia could not induce autophagy in Park2 KO mice. Parkin protein was decreased in the spinal cord in Park2 KO mice (Figures 7(e) and 7(f)), but the HIF-1*α* level was not changed in the spinal cord in Park2 KO mice compared to WT mice (Figures 7(g) and 7(i)). We explored whether HIF-1*α* agonist DMOG could induce mitophagy in Park2 KO diabetic mice. LC3-II, Beclin1, and P62 proteins did not change in Park2 KO diabetic mice after DMOG treatment (Figures 7(a)–7(d)). These results were verified by the immunofluorescence double-labelling technique. The number of colocalization of LC3-II and TOM20 cells was higher in Park2 WT diabetic mice than in Park2 KO diabetic mice (Figure 7(i)). Moreover, the number of colocalization cells could not be increased by DMOG treatment in Park2 KO diabetic mice (Figure 7(i)). Otherwise, the level of HIF-1*α* was increased by DMOG in both Park2 KO and WT diabetic mice (Figures 7(g) and 7(h)). These findings suggested that mitophagy could not be induced and upregulated by HIF-1*α* in Park2 KO mice. Mitochondrial autophagosomes were induced by hyperglycemia in WT mice, but not in the Park2 KO mice (Figure 7(j)).

## 4. Discussion

Mitochondrial dysfunction, induced by hyperglycemia, was considered a key mediator in the pathogenesis of DNP and other diabetes-related complications. Therefore, improving mitochondrial dysfunction would be a promising therapeutic strategy for the treatment of DNP. In this study, we found that upregulation of HIF-1*α* could improve mitochondrial dysfunction and increase mitophagy and alleviate hyperalgesia in WT diabetic mice, but not in Park2-deficient diabetic mice. These results indicated that HIF-1*α* alleviated hyperalgesia through Parkin-mediated mitophagy.

Recently, studies have demonstrated that mitochondrial contributed to sensory processing and induced neuropathic pain, including diabetic neuropathic pain [45, 46]. Since mitochondrial dysfunction was the key factor in the induced DNP, mitophagy, which can improve mitochondrial dysfunction and prevent excessive ROS generation, may be a promising therapeutic treatment for neuropathic pain. To our knowledge, we found for the first time that mitophagy in the spinal cord increased in STZ-induced diabetic mice. Mitophagy was a major approach to controlling mitochondrial quality by removing damaged mitochondria and inhibiting oxidative stress [47]. However, the change in mitophagy was not consistent with diabetes-related complications. Zhou et al. demonstrated that mitophagy was degreased in podocytes, and restored mitophagy could reduce renal injury in diabetic mice [19]. Conversely, mitophagy was increased in the diabetic heart, and it could inhibit diabetic cardiomyopathy. Although the mitophagy levels in the diabetic heart and kidney were different, increased mitophagy can alleviate diabetic heart and kidney injury.

In the present study, we found that ROS accumulation and decreased mitochondrial membrane potential occurred in the spinal cord of diabetic mice. Overexpression of HIF-1*α* could improve mitochondria dysfunction and increase mitophagy. Otherwise, inhibition of HIF-1*α* decreased mitophagy induced by hyperglycemia and aggravated mitochondrial dysfunction. These results suggest that mitophagy caused by hyperglycemia was an intracellular protection mechanism in diabetic mice. Similarly to our study, previous studies have shown that increased mitophagy could alleviate nerve injury-induced neuropathic pain [17, 40]. HIF-1*α* is a key subunit of hypoxia-inducible factor 1 (HIF-1), and it is a critical regulatory molecule when the cell is under hypoxic. Under normal oxygen conditions, HIF-1*α* can be hydroxylated by proline-4-hydroxylase domain-containing enzyme (PhD), then linked by E3 ubiquitin ligase, and finally recognized and degraded by the proteasome. Under hypoxia, intracellular PhD activity was inhibited and HIF-1*α* could not be hydroxylated in time. Then, HIF-1*α* was translocated into the nucleus and combined to HIF-1*β* to form an active HIF-1 complex which can regulate downstream gene transcription. This study showed that HIF-1*α* was activated in the spinal cord of diabetic mice, and similar results were reported in the heart, retina, and kidney tissue in diabetic animals [27]. However, the function of HIF-1*α* in different organs of diabetic animals may be other. Increased HIF-1*α* level played a protective role in the diabetic heart and kidney [27] but aggravated diabetes retinopathy. Therefore, the function of HIF-1*α* in different diabetic complications should be further explored. Recent research suggested that HIF-1*α* was increased in peripheral nerve fibers in patients with diabetes [29], and it implied the relationship between HIF-1*α* and diabetic peripheral neuropathy. In our study, the expression of HIF-1*α* was increased and its agonist DMOG can alleviate hyperalgesia. It indicated that HIF-1*α* could play a protective role in DNP. Consistent with the results of our study, Kanngiesser et al. have shown that HIF-1*α*^−/−^mice were more susceptible to noxious cold and hot pain stimulation, and indicated HIF-1*α* has a protection function in pain [48]. A recent study also demonstrated that overexpression of HIF-1*α* could attenuate hyperalgesia in rats following chronic constriction injury [47]. Moreover, the mitophagy induced by hyperglycemia can be further induced by HIF-1*α* agonist DMOG but inhibited by HIF-1*α* antagonist. These results revealed that HIF-1*α* exerted a protective effect against mitochondrial dysfunction in diabetic mice, which could be mediated via increased mitophagy. An existing question is why the expression of HIF-1*α* was elevated in the diabetic mice when it has a protective effect on DNP. The overexpression and activity of HIF-1*α* may be one of the compensatory responses to hyperglycemia-related injury.

To further explore the mechanism of HIF-1*α*-regulated mitophagy in DNP, we knock out the Park2 gene, which encodes Parkin was an important regulator of mitophagy. Mitochondrial depolarization by various stimuli is a common trigger for mitophagy. When mitochondria membrane potential was decreased, phosphatase and tensin homolog-induced putative kinase 1 (PINK1) becomes shifted and stabilized on the dysfunction mitochondrial outer membrane [49]. The activated PINK1 then recruited Parkin to depolarize mitochondria [49] and then further connected with p62 and LC3 for ubiquitination degradation [50, 51]. Recently, a study reported that Parkin could eliminate the impaired mitochondria through mitophagy in PD. In addition, Park2 gene mutations lead to Parkin deficiency, which induced oxidative stress and mitochondrial dysfunction [52]. In our study, we found that Parkin was increased in the spinal cord of diabetic mice, complied with increased mitophagy. Otherwise, the mitophagy could not be induced in Parkin-deficient diabetic mice. These results suggest that hyperglycemia-induced mitophagy depends on the Parkin protein. In addition, the expression of HIF-1*α* was increased in both Park2 WT and KO diabetic mice, but MMP loss and ROS accumulation were significantly reduced by the specific HIF-1*α* agonist in Park2 WT mice but not in Park2 KO mice. Collectively, our data described herein showed that HIF-1*α* increased mitophagy and improved mitochondrial dysfunction involved in Parkin in diabetic mice.

There are several limitations to this study. First, mitophagy is a dynamic process, and we only detected mitophagy on five weeks after STZ injection, which may have certain limitations. But we found HIF-1*α* agonists and inhibitors could regulate mitophagy and hyperalgesia in WT mice but not in Park2 KO mice, which demonstrated mitophagy could regulation DNP. To further clarify the dynamic changes in the mitophagy process, we should observe multiple time points. Second, ideal mitophagy monitoring should be included both autophagosome and lysosome markers to colocalize and monitor this dynamic process. However, the overwhelming majority of studies only detect autophagosome markers and are considered sufficient to respond to changes in autophagy. Finally, mitochondrial membrane potential and ROS production were the main mediators but were not completely representative of mitochondrial function. There were some other indicators, including ATP levels, respiratory function, and intracellular calcium ion levels, related to mitochondrial function which should be monitored in future experiments.

## 5. Conclusions

The conclusion of the present study is that HIF-1*α* could alleviate diabetic neuropathic pain through mitophagy. In addition, the function of HIF-1*α* regulate mitophagy depends on Parkin protein. Consequently, our study improves the understanding of HIF-1*α* and Parkin-mediated mitophagy and provides the scientific basis for the use of HIF-1*α* and mitophagy as potential therapeutic targets in the clinical management of in DNP.

## Figures and Tables

**Figure 1:** Overexpression of HIF-1*α* of the spinal cord in diabetic mice. (a, b) Western blot analysis, the level of HIF-1*α*. (c, d) Immunohistochemical analysis of the level of HIF-1*α* in the spinal cord. The red arrows indicated the HIF-1*α*-positive cells. ^a^*P* < 0.05 vs. NC; ^b^*P* < 0.05 vs. DP. NC: control mice group; DP: diabetic mice group; ME: diabetic mice group administered methoxyestradiol (2-ME, HIF-1*α* inhibitor); DM: diabetic mice group administered dimethyloxalylglycine (DMOG, HIF-1*α* agonist).

**Figure 2:** Overexpression of HIF-1*α* alleviate hyperalgesia in diabetic mice. (a) The blood glucose changes after streptozotocin (STZ) injection, (b) the paw withdrawal threshold (PWT) change of mice after STZ and HIF-1*α* agonist or antagonist injection, and (c) thermal withdrawal latency (TWL) change of mice after STZ and HIF-1*α* agonist or antagonist injection. ^#^*P* < 0.05 vs. NC; ^∗^*P* < 0.05 vs. DP. NC: control mice group; DP: diabetic mice group; ME: diabetic mice group administered 2-ME (HIF-1*α* inhibitor); DM: diabetic mice group administered DMOG (HIF-1*α* agonist).

**Figure 3:** Overexpression of HIF-1*α* improved mitochondrial dysfunction in the spinal cord of diabetic mice. (a) Mitochondrial membrane potential detection by flow cytometry analysis using JC-1, Q1-UR/LR ration was indicated JC-1 aggregates/monomer ratio and analyzed by statistic. (b) ROS content detection by flow cytometry analysis using 2′,7′-dichlorofluorescein diacetate. ^a^*P* < 0.05 vs NC; ^b^*P* < 0.05 vs DP. NC: control mice group; DP: diabetic mice group; ME: diabetic mice group administered 2-ME (HIF-1*α* inhibitor); DM: diabetic mice group administered DMOG (HIF-1*α* agonist).

**Figure 4:** Overexpression of HIF-1*α* increased mitophagy in the spinal cord of diabetic mice. (a) The level of autophagy marker LC3, Beclin1, and P62 in the spinal cord by western blot examination. (b) Expression of TOM 20 and LC3 in the spinal dorsal horn using double-immunolabeled. (c) Mitochondrial autophagosome in the spinal cord by electron microscope. ^a^*P* < 0.05 vs. NC; ^b^*P* < 0.05 vs. DP. NC: control mice group; DP: diabetic mice group; ME: diabetic mice group administered 2-ME (HIF-1*α* inhibitor); DM: diabetic mice group administered DMOG (HIF-1*α* agonist).

**Figure 5:** Park2 deficiency accelerated the development of neuropathic pain in diabetic mice. (a) The blood glucose concentration in Park2 knockout (KO) and wild-type (WT) mice after STZ injection, (b–d) the PWT change in Park2 KO and WT diabetic mice after STZ and drug injection, and (e–g) the TWL change in Park2 KO and WT diabetic mice after STZ and drugs injection. ^#^*P* < 0.05 vs. WT+NC or KO+NC; ^∗^*P* < 0.05 vs. WT+DP or KO+DP. NC: control mice group; DP: diabetic mice group; DM: diabetic mice group administered DMOG (HIF-1*α* agonist).

**Figure 6:** Park2 knockout aggravated mitochondrial dysfunction in the spinal cord of diabetic mice. (a, b) ROS content detection by flow cytometry analysis using 2′,7′-dichlorofluorescein diacetate, (c, d) Mitochondrial membrane potential detection by flow cytometry analysis using JC-1, Q1-UR/LR ration was indicated JC-1 aggregates/monomer ratio and analyzed by statistic. ^a^*P* < 0.05 vs. WT+NC; ^b^*P* < 0.05 vs. WT+DP. ^C^*P* < 0.05 vs. KO+NC; NC: control mice group; DP: diabetic mice group; DM: diabetic mice group administered DMOG (HIF-1*α* agonist).

**Figure 7:** Mitophagy could not be induced by hyperglycemia in the spinal cord in Parkin-deficient mice. (a–d) The expression of LC3, Beclin1, and P62 in the spinal cord of Park2 KO and WT mice using western blot. (e, f) The expression of Parkin in the spinal cord of Park2 KO and WT mice using western blot. (g, h) The expression of HIF-1*α* in the spinal cord of Park2 KO and WT mice using western blot. (i) Expression levels of Tom 20 and LC3 in the spinal dorsal horn using double-immunolabeled, (j) Mitochondrial autophagosome in the spinal cord using electron microscope. ^a^*P* < 0.05 vs. WT+NC; ^b^*P* < 0.05 vs. WT+DP; ^C^*P* < 0.05 vs. KO+NC; ^d^*P* < 0.05 vs. KO+DP. NC: control mice group; DP: diabetic mice group; DM: diabetic mice group administered DMOG (HIF-1*α* agonist).

## Data Availability

The data used to support the findings of this study are available from the corresponding author upon request.
